# Stent patency rates and prognostic factors of endovascular intervention for iliofemoral vein occlusion in post-thrombotic syndrome

**DOI:** 10.1186/s12893-022-01714-9

**Published:** 2022-07-12

**Authors:** Rencong Chen, Ruijia Feng, Suiting Jiang, Guangqi Chang, Zuojun Hu, Chen Yao, Benyuan Jia, Shenming Wang, Siwen Wang

**Affiliations:** 1 Division of Vascular Surgery, The First Affiliated Hospital, Sun Yat-Sen University, No. 58, Zhongshan 2nd road, Yuexiu District, Guangzhou, 510080 Guangdong China; 2 Guangdong Engineering Laboratory of Diagnosis and Treatment of Vascular Disease, Guangzhou, 510080 China

**Keywords:** Post-thrombotic syndrome, Endovascular intervention, Iliofemoral vein, Iliofemoral stent, Patency rate

## Abstract

**Objective:**

Post-thrombotic syndrome (PTS), an important complication of deep venous thrombosis (DVT), adversely affects patients’ quality of life. Endovascular intervention in PTS can relieve symptoms rapidly with high therapeutic value. This study mainly focuses on how to improve postoperative stent patency rates and aims to find prognostic factors impacting patency.

**Methods:**

According to the specific inclusion and exclusion criteria, PTS patients who underwent endovascular intervention at the First Affiliated Hospital of Sun Yat-sen University from December 1, 2014, to December 31, 2019, were included in this single-center prospective study. Follow-up data were collected and analyzed regularly over 2 years.

**Results:**

Overall, 31 PTS patients were enrolled in the study. The mean age of these patients was 55.39 ± 11.81, including 19 male patients. Stent implantation was successful in 22 PTS patients, with a technical success rate of 70.97%. The average Villalta scores of the stent-implanted group and the non-stent-implanted group were 5.95 ± 2.57 and 5.78 ± 2.95, respectively, with no significant difference observed. In the stent-implanted group, the perioperative patency rate was 81.81% (18/22), and the follow-up patency rates were 68.18% (15/22) within 3 months, 59.09% (13/22) within 6 months, 45.45% (10/22) within 1 year, and 36.36% (8/22) within 2 years. Based on the stent placement segments, the 22 PTS patients were divided into two subgroups: the iliofemoral vein balloon dilation + iliofemoral vein stent implantation (FV-S) subgroup and the iliofemoral vein balloon dilation + iliac vein stent implantation (FV-B) subgroup. In the FV-S subgroup, the perioperative patency rate was 100.00% (14/14), and the follow-up patency rates were 85.71% (12/14), 71.43% (10/14), 57.14% (8/14) and 50.00% (7/14), which were higher than those for overall stent patency of all patients. The postoperative patency rates in the FV-B subgroup were 50.00% (4/8), 37.50% (3/8), 37.50% (3/8), 25.00% (2/8), and 12.50% (1/8). The secondary postoperative patency rates in the FV-B subgroup were 100.00% (8/8), 87.50% (7/8), 75.00% (6/8), 62.50% (5/8) and 50.00% (4/8).

**Conclusions:**

For PTS patients with iliofemoral vein occlusion but patent inflow, iliofemoral vein stent implantation is a more efficient therapeutic option than iliofemoral vein balloon dilation with iliac vein stent implantation for PTS patients.

## Introduction

Post-thrombotic syndrome (PTS) is a kind of complication that adversely affects the quality of life of deep venous thrombosis (DVT) patients. The venous hypertension which is the pathophysiological factor caused by continuous occlusion of venous return contributes to the development of PTS, which would further present special symptoms or signs such as pain, varicose veins, swelling of limbs, pigmentation and keratinization of skin, ulcer formation as well as paresthesia [1]. PTS is mainly treated with compression treatment (usually elastic compression stockings) to relieve symptoms [2]. Endovascular balloon dilation and stent implantation can open iliofemoral vein occlusion in PTS patients and relieve symptoms quickly, so it has high therapeutic value [3–7]. However, previous studies indicated that both the short-term and patency rates of endovascular intervention in PTS patients were relatively low, and the risk of in-stent restenosis or reocclusion might not be acceptable, limiting the application of this procedure [8–11]. Thus, the indications and patient candidates for endovascular intervention should be considered carefully [12]. This study aims to explore how to expand the indications for endovascular intervention and increase the short-term and patency rates in PTS patients. In addition, we summarize optimal methods and our clinical experience to improve the outcome and prognosis of endovascular intervention in PTS patients.

## Method

### Patient selection

This is a prospective study based on all PTS patients who were admitted to the First Affiliated Hospital of Sun Yat-sen University from December 1, 2014, to December 31, 2019. The main inclusion criteria were as follows: (1) DVT history and ipsilateral lower limb deep venous insufficiency based on imaging examination; (2) relevant interventional procedures for PTS; (3) according ultra-sound or computer tomography, at least femoral vein or/and profunda femoris vein has patent inflow (stenosis < 50%). This study followed the Strengthening the Reporting of Observational Studies in Epidemiology (STROBE) reporting guideline. Ethics approval (Approval number:2013C-193) for this study was obtained from the ICE for Clinical Research and Animal Trial of the First Affiliated Hospital of Sun Yat-sen University at the commencement of this study. All the participants signed formal informed consent to participate in this study and their information was well protected.

### Intervention

The procedures were all performed under local anesthesia. Under ultrasound guidance, we punctured ipsilateral femoral vein, popliteal vein, great saphenous vein, or tibiofibular trunk to establish vascular access, followed by anticoagulation with heparin sodium. Once the wire and the catheter went through the occlusion lesion to inferior vena cava, catheter will be switched to balloons with appropriate diameters which will be gradually inflated. And then stents were strictly selected according to the distal and proximal diameter of the relevant veins, and the placement of the distal end of the stent across the hip joint was avoided as much as possible during the primary intervention [11]. After stent implantation, adequate anticoagulant therapy for preventing in-stent thrombosis will be conducted throughout the follow-up period. The secondary intervention was mainly in-stent catheter-directed thrombolysis or pharmaco-mechanical thrombectomy combined with balloon dilation and extending stent implantation at the distal end of the former iliac vein stent.

### Statistical variables

We collected a large number of variables, such as patient characteristics, information on surgical procedures, perioperative condition and follow-up data (the variables are shown in Tables 1, 2, 3). Patient characteristics included sex, age, complications, duration of symptoms, duration since DVT onset, Clinical-Etiology-Anatomy-Pathophysiology (CEAP) grade, Villalta score, PTS severity (ulcer condition) and preoperative imaging examination results (color Doppler ultrasonography and computed tomography). Surgical procedures included the time of intervention, puncture site, whether the occluded segment was successfully passed, number of balloons, brand and number of stents. The surgical procedures were divided into iliofemoral vein balloon dilation + iliofemoral vein stent implantation (FV-S) and iliofemoral vein balloon dilation + iliac vein stent implantation (FV-B) according to the segment of the stent (whether placed in the common femoral vein or femoral vein). Perioperative conditions included postoperative complications, stent patency, and information on preoperative and postoperative anticoagulant therapy. Follow-up data included the Villalta score, PTS severity (ulcer condition), incidence of restenosis or reocclusion after stent implantation, postoperative patency rates within 1 month/3 months/6 months/1 year/2 years, and secondary intervention procedures.

**Table 1:** Patient characteristics of stent-implanted group and the non-stent-implanted group

Variable	Stent-implanted group	Non-stent-implanted group	P value
No. of cases	22	9	
Mean age	54.23 ± 11.21	58.22 ± 13.41	0.402
Duration of symptoms (month)	51.39(0.5–360)	45.67(6–120)	0.838
Duration of DVT onset (month)	84.05(5–360)	46(6–120)	0.214
Preoperative Villalta score	5.95 ± 2.57	5.78 ± 2.95	0.869
PTS severity (ulcer condition)	10/22	4/9	0.959
Preoperative long-term anticoagulant therapy	10/22	5/9	0.609

DVT: deep venous thrombosis; PTS: post-thrombotic syndrome

**Table 2:** Patient characteristics, postoperative PTS symptoms, perioperative conditions, deep vein anatomic conditions, surgery procedures and postoperative patency rates in 22 PTS patients

Patient#	Time of surgery	Duration of symptoms (month)	Duration of DVT onset (month)	CEAP	Villalta score	PTS severity	Short-term postoperative Villalta score	Ulcer	preoperative anticoagulant drug	postoperative anticoagulant drug	Stenosis and occlusion severity (%)						Access veins	Location of balloon dilation	Location of stents placement	Postoperative patency				
											CIV	EIV	CFV	FV	PFV	PV				1 m	3 m	6 m	12 m	24 m
1	2014/12/9	120	120	C5	6	Mild	6	0	0	Warfarin	100	100	70–80	50	0	50	LFV	LCIV, LEIV, LCFV	LCIV, LEIV, LCFV	P	P	P	P	P
2	2015/5/26	12	120	C2	4	Mild	4	0	Warfarin	Rivaroxaban	100	100	0	0	0	0	LFV	LCIV, LEIV	LCIV, LEIV, LCFV	P	P	P	P	P
3	2015/8/11	36	144	C6	7	Severe	6	Unhealed	Warfarin	Warfarin	< 50	100	< 50	< 50	< 50	< 50	RFV	RCIV, REIV	RCIV, REIV, RCFV	P	O(P)^a^	O(P)	O(P)	O(P)
4	2016/1/12	4	10	C4	7	Mild	6	0	0	Warfarin	< 50	< 50	< 50	< 50	< 50	< 50	LGSV	LCIV, LEIV, LCFV	LCIV, LEIV, LCFV	P	P	P	P	P
5	2016/5/4	0.5	60	C4	5	Mild	3	0	Warfarin	Warfarin	100	0	0	0	0	0	LFV	LCIV, LEIV	LCIV, LEIV	O(P)	O(P)	O(P)	O(P)	O(P)
6	2016/5/6	18	18	C3	5	Mild	4	0	Rivaroxaban	Rivaroxaban	100	100	0.5–0.69	100	50–69	0	LFV	LCIV, LEIV	LCIV, LEIV	O(P)	O(O)	O(O)	O(O)	O(O)
7	2016/5/25	3	24	C4	6	Mild	4	0	Warfarin	Warfarin	< 50	100	< 30	40–60	0	40–60	RPV	RCIV, REIV, RCFV	RCIV, REIV, RCFV	P	P	P	P	P
8	2016/7/26	24	24	C1	1	Mild	1	0	Rivaroxaban	Rivaroxaban	100	100	< 50	0	0	0	LPV	LCIV, LEIV, LCFV	LCIV, LEIV	O(P)	O(P)	O(P)	O(P)	O(P)
9	2016/11/1	120	120	C6	3	Severe	2	Unhealed	0	Rivaroxaban	0	100	< 50	0	0	0	LPV	LCIV, LEIV, LCFV	LCIV, LEIV, LCFV	P	P	P	P	P
10	2016/12/16	12	12	C4	5	Mild	2	0	Rivaroxaban	Rivaroxaban	100	0	0	100	0	0	LPV	LCIV, LEIV, LCFV	LCIV, LEIV, LCFV	P	P	P	P	P
11	2017/1/10	24	24	C4	5	Mild	2	0	0	Rivaroxaban	50	50	0	0	0	0	LPV	LCIV, LEIV, LCFV	LCIV, LEIV, LCFV	P	O(O)	O(O)	O(O)	O(O)
12	2017/2/21	5	5	C6	7	Severe	7	Healed	0	Warfarin	< 50	0	< 50	< 50	0	0	LPV	LCIV, LEIV	LCIV, LEIV, LCFV	P	P	P	P	P
13	2017/6/15	48	60	C6	10	Severe	8	Healed	0	Rivaroxaban	< 50	< 50	< 50	< 50	0	< 50	LFV	LCIV, LEIV	LCIV, LEIV	P	P	P	P	O
14	2017/6/29	96	228	C6	7	Severe	5	Healed	0	Warfarin	100	100	50	0	0	0	Left tibiofibular trunk	LCIV, LEIV	LCIV, LEIV	P	P	P	O	O
15	2017/8/22	1	14	C3	2	Mild	2	0	Rivaroxaban	Rivaroxaban	100	0	0	0	0	0	LPV	LCIV, LEIV	LCIV, LEIV	O(P)	O(P)	O(P)	O(P)	O(P)
16	2018/3/12	4	84	C6	2	Severe	2	Healed	0	Rivaroxaban	50	100	30–40	60–70	0	60–70	RPV	RCIV, REIV, RCFV	RCIV, REIV, RCFV	P	P	P	P	O
17	2018/5/3	60	110	C6	10	Severe	8	Recurrent	0	Rivaroxaban	100	100	50–69	0	0	0	LPV	LCIV, LEIV, LCFV	LCIV, LEIV, LCFV	P	P	P	O(P)	O(P)
18	2018/6/19	12	12	C5	8	Mild	6	0	0	Rivaroxaban	100	100	0	0	0	0	LPV	LCIV, LEIV	LCIV, LEIV	P	P	P	P	P
19	2018/7/9	72	72	C4	10	Moderate	8	0	Warfarin	Rivaroxaban	100	100	50–75	50–100	0	< 50	LPV, RCFV	LCIV, LEIV	LCIV, LEIV, LCFV	P	P	O(P)	O(O)	O(O)
20	2018/10/23	3	60	C6	9	Severe	7	Healed	0	Rivaroxaban	100	100	60–70	100	0	100	LGSV	LCIV, LEIV	LCIV, LEIV, LCFV	P	P	O	O	O
21	2019/3/25	96	168	C6	6	Severe	6	Healed	0	Rivaroxaban	70–100	70–100	70–100	70–100	0	70–100	LPV	LCIV, LEIV, LCFV	LCIV, LEIV, LCFV	P	P	P	O(O)	O(O)
22	2019/9/16	360	360	C6	6	Severe	5	Healed	Rivaroxaban	Rivaroxaban	100	100	100	100	0	0	LPV	LCIV, LEIV, LCFV	LCIV, LEIV	P	O(P)	O(O)	O(O)	O(O)

CIV: common iliac vein; EIV: external iliac vein; CFV: common femoral vein; FV: femoral vein; PFV: profunda femoris vein; PV: popliteal vein; LCIV: left common iliac vein; RCIV: right common iliac vein; LEIV: left external iliac vein; REIV: right external iliac vein; LCFV: left common femoral vein; RCFV: right common femoral vein; LFV: left femoral vein; RFV: right femoral vein; LPV: left popliteal vein; RPV: right popliteal vein; LGSV: lift great saphenous vein; PTS: post-thrombotic syndrome; CEAP: Clinical-Etiology-Anatomy-Pathophysiology; m: months; P: patent; O: occlusion

^a^Patency outcome of re-intervention

**Table 3:** Factors associated with perioperative stent patency rate in PTS patients

Variable	perioperative stent patency	perioperative re-occlusion	P value
No. of cases	18	4	
Duration of symptoms (month)	63.39(3–360)	10.88(0.5–24)	0.271
Duration of DVT onset (month)	92.28(5–360)	29.00(14–29)	0.163
Villalta score	6.56 ± 2.31	3.25 ± 2.06	0.016
CEAP grade (C4, C5, C6)	17/18	1/4	0.001
PTS severity (ulcer condition)	10/18	0/4	0.044
Preoperative long-term anticoagulant therapy	6/18	4/4	0.015
Postoperative long-term anticoagulant therapy (warfarin)	6/18	1/4	0.350

DVT: deep venous thrombosis; PTS: post-thrombotic syndrome; CEAP: Clinical-Etiology-Anatomy-Pathophysiology

### Outcomes and definitions

The primary outcome was the primary patency rate. And secondary outcome was the secondary patency rate. The perioperative patency rate was defined as the stent patency rate within 1 month after intervention, while the follow-up patency rate was defined as the stent patency rate from the 1 month to 2 years after intervention. The patency rates were evaluated by computed tomography angiography (CTA) or intravascular ultrasound (IVUS).According to the Society of Vascular Surgery standard, primary patency rate was defined as absence of stent occlusion without additional or secondary surgical or endovascular procedures.. Secondary patency rate was defined as the proportion of patients who maintained stent patency after an additional or secondary surgical or endovascular procedure after stent occlusion [13–15].

### Statistical analysis

All statistical analyses were performed using SPSS Statistics version 26 and R software (v.4.0.1, https://www.r-project.org/about.html). The rates of events were calculated as the number of events divided by the number of treated patients with available data. The results were presented as the median ± IQR or ranges as appropriate. Comparisons between the patients in different groups or subgroups were made using Fisher's exact test for categorical variables and a Mann–Whitney U test for continuous variables. Kaplan–Meier survival curves with log-rank analyses were created to assess the cumulative primary and secondary patency rates. The 95% confidence intervals (CIs) for the patency rates were calculated. A P value of < 0.05 was considered statistically significant.

## Results

Thirty-one PTS patients underwent relevant interventional procedure at the First Affiliated Hospital of Sun Yat-sen University from December 1, 2014, to December 31, 2019 (Fig. 1). The mean age of these patients was 55.39 ± 11.81, including 19 male patients. Of all patients undergoing interventional procedure, the guide wire and catheter failed to pass through the occlusive segment in 9 PTS patients, and endovascular intervention was successfully performed in 22 PTS patients. The patient characteristics of the two groups are shown in Table 1. The mean ages of the stent-implanted group and the non-stent-implanted group were 54.23 ± 11.21 years and 58.22 ± 13.41 years, respectively, with no significant difference observed. The average Villalta scores of the two groups were 5.95 ± 2.57 and 5.78 ± 2.95, respectively, with no significant difference observed. There were also no significant differences between the two groups in terms of the duration of symptoms, duration since DVT onset, PTS severity or preoperative anticoagulant therapy.

**Fig. 1:** Diagram of the data collection process

Among the 22 PTS patients in the stent-implanted group, the perioperative patency rate was 81.81% (18/22). Color Doppler ultrasonography before discharge (within 1 week after the operation) suggested reocclusion in 4 PTS patients, so reintervention was performed. The overall deep vein anatomic conditions (stenosis or occlusion greater than or equal to 50%) with concomitant surgical procedures and postoperative patency rates are shown in Table 2. The 4 PTS patients with reocclusion were all patients whose stents were not placed at the common femoral vein or femoral vein. In addition, there was a certain difference in the perioperative and follow-up patency rates between the two procedures (Fig. 2). The perioperative patency rate was 50% (4/8) in the patients in the FV-B subgroup but 100% (14/14) in the patients in the FV-S subgroup. The primary follow-up patency rates of patients in FV-S subgroup were 85.71% (12/14), 71.43% (10/14), 57.14% (8/14) and 50.00% (7/14) within 3 months, 6 months, 1 year and 2 years, respectively, which were higher than the overall patency rates of all follow-up patients, namely, 68.18% (15/22), 59.09% (13/22), 45.45% (10/22), 36.36% (8/22), respectively, and were also significantly higher than those of patients in FV-B (P < 0.05, Fig. 2), namely, 37.50% (3/8), 37.50% (3/8), 25.00% (2/8), and 12.50% (1/8), respectively. Reocclusion occurred in patient No. 8 during the perioperative period because the common femoral vein was not efficiently dilated by the balloon and the stents were not placed. During hospitalization, the common femoral vein was reinflated by a balloon, and stents were implanted. During follow-up, no stent occlusion was found. Meanwhile, with concomitant femoral vein stenosis or occlusion (stenosis > 50%), profunda femoris vein stenosis might impact the perioperative and follow-up patency rates. As shown in Table 2, patients No. 6 and No. 3 had different degrees of profunda femoris vein stenosis. Perioperative and postoperative reocclusion (at the third month of follow-up) were observed. Patient No. 6 experienced reocclusion once again a short period after reintervention. After iliofemoral vein balloon dilation + iliac vein stent implantation, the secondary patency rates during the perioperative period and follow-up period were significantly increased to 100.00% (8/8), 87.50% (7/8), 75.00% (6/8), 62.50% (5/8) and 50.00% (4/8), respectively, after the secondary intervention (common femoral vein or femoral vein stent implantation).

**Fig. 2:** The primary (**A**, **C**) and secondary (**B**, **D**) stent patency rates within the 12-month and 24-month follow-up examination in two subgroups respectively. The tabular data present the number of patients

Eighteen PTS patients with perioperative stent patency were compared with 4 PTS patients who experienced perioperative reocclusion (Table 3). There was no significant difference in the duration of symptoms, duration since DVT onset or postoperative anticoagulant therapy between the two subgroups. However, the preoperative Villalta score of the patients with perioperative reocclusion was significantly lower than that of the patients with perioperative patency (P = 0.016), which was consistent with the CEAP grade (proportion of patients with C4, C5 and C6) (P = 0.001). The PTS severity (ulcer condition) in the reocclusion subgroup was also significantly lower than that in the patency subgroup (P = 0.044). In addition, in terms of preoperative anticoagulant therapy, the patency group required significantly less therapy than the reocclusion group (P = 0.015).

## Discussion

In this study, the prognostic factors impacting patency were analyzed in PTS patients treated with interventional procedures at a single center over the past 5 years. According to the comparison between the stent-implanted group and the non-stent-implanted group, we suggested that PTS severity, the duration of symptoms or the duration of DVT onset had no correlation with the success of intervention. Preoperative anticoagulation therapy also showed little influence on surgical success. Therefore, it is difficult to determine whether a PTS patient meets the indications for endovascular intervention if considering only past medical history and preoperative ultrasound or CT.

Another effective indicator of the therapeutic outcome of endovascular intervention is the postoperative primary patency rate. In this study, the overall perioperative patency rate was 81.8%, but the two-year follow-up patency rate was less than 40%. Compared to other centers, the patency rate was only 51.75% within 30 days after intervention, and the two-year follow-up patency rate was only 38.18%. Therefore, the overall postoperative patency rates for PTS patients may not be relatively high [11, 16–18]. However, data from our center and other studies [11] have revealed that endovascular intervention can lead to significant improvement in PTS symptoms (Villalta score [19]) and signs (ulcer condition). Therefore, how to improve the postoperative patency rates in endovascular intervention deserves further study.

Previous studies have indicated that it is necessary to ensure enough capacity and speed of blood inflow in iliofemoral stents to reduce the incidence of reocclusion or thrombosis [20]. Therefore, evaluation of venous inflow is obviously important. Our study also verified that it is difficult to maintain stent patency with concomitant obstructed profunda femoris veins. By analyzing the surgical procedures of 4 PTS patients with perioperative reocclusion, we found that all of them underwent iliofemoral vein balloon dilation + iliac vein stent implantation; Further analysis suggested that, for patients No. 5 and No. 15 in Table 2, the lesion only involved the common iliac vein, so endovascular intervention was only performed in the common iliac vein and external iliac vein. However, perioperative reocclusion occurred in both cases. Therefore, we speculated that the perioperative and follow-up patency rates of PTS patients are closely correlated with surgical procedures, which is further illustrated in Table 3. The perioperative and follow-up patency rates of patients after iliofemoral vein balloon dilation + iliofemoral vein stent implantation were higher than the overall patency rate of all patients completing follow-up. However, the perioperative and patency rates of patients after iliofemoral vein balloon dilation + iliac vein stent implantation were decreased. This may be because PTS patients tend to develop more collateral branches, which originate from the opening of the profunda femoris vein or the common femoral vein to the inferior vena cava. Balloon dilation of the common femoral vein can increase iliofemoral vein blood inflow and simultaneously reduce collateral blood flow. In addition, the openings of collateral branches on the common femoral vein were covered by the stents to a certain extent, which could produce the same effect. Consequently, patent blood inflow appeared after iliofemoral vein balloon dilation + iliofemoral vein stent implantation. However, this conclusion is controversial in some published studies. Relevant studies have found that for severe PTS patients with normal profunda femoris veins complicated with iliofemoral lesions, iliofemoral vein balloon dilation + iliofemoral vein stent implantation cannot improve the stent patency rate [11].

Moreover, previous studies have shown that the stent type, design, texture and so on have a certain effect on stent patency. When the same PTS severity and stent was analyzed, it was found that whether the stent is placed across the joints (hip joint) may also affect patency rates [5, 21–23].

## Limitations

The current study describes how to improve postoperative stent patency rates and aims to find the prognostic factors impacting patency in severe PTS patients. However, the results of this study require further validation by evaluating more cases in comparisons of the FV-S subgroup and FV-B subgroup. On the other hand, prospective multicenter registry data can provide more accurate data. Moreover, the study was nonrandomized, and it may have obvious selection bias. Therefore, further randomized studies are still needed to validate these conclusions.

## Conclusion

For PTS patients with iliofemoral vein occlusion but patent inflow, the patency rates after endovascular intervention showed no significant correlations with patient characteristics or long-term preoperative anticoagulant therapy. Endovascular intervention can improve PTS symptoms, lower the incidence of limb ulcers and improve patient quality of life to a certain extent. Endovascular intervention appears to relieve PTS symptoms and improve limb venous ulcer healing. With patent inflow, iliofemoral vein stent implantation is an efficient treatment for PTS patients.

## Data Availability

All data generated or analyzed during this study are included in this article.

## Abbreviations

PTS: Post-thrombotic syndrome
DVT: Deep venous thrombosis
FV-S: Iliofemoral vein balloon dilation + iliofemoral vein stent implantation
FV-B: Iliofemoral vein balloon dilation + iliac vein stent implantation
CEAP: Clinical-Etiology-Anatomy-Pathophysiology
CI: Confidence interval
